The article "Comparison of the Effects of Laparoscopic Surgery and Traditional Open Surgery on Stone Clearance, Laboratory Indexes and Life Quality in Patients with Renal Calculi" was retracted in 2023. Reasons: signs of a paper mill; compromised peer review; unreliable results or conclusions.

# Comparison of the Effects of Laparoscopic Surgery and Traditional Open Surgery on Stone Clearance, Laboratory Indexes and Life Quality in Patients with Renal Calculi

**DOI:** 10.1155/2022/8211389

**Published:** 2022-09-29

**Authors:** Qian Ai, Dong Tang, Yongfa Li, Yingjie Huang, Junxian Yang

**Affiliations:** ^1^Department of Urology, Wuhan Puren Hospital, No. 1 Benxi street, Qingshan District, Wuhan City, Hubei Province 430081, China; ^2^Tianyou Hospital Affiliated to Wuhan University of Science and Technology, 430064, China

## Abstract

**Objective:**

A case-control study was conducted to determine the effectiveness of laparoscopic surgery and traditional open surgery on stone clearance, laboratory indexes, and life quality in patients with renal calculi.

**Methods:**

During March 2017 to March 2022, 272 patients with complex renal calculi (CRC) cured in our hospital were assigned into control group (*n* = 136) and research group (*n* = 136) arbitrarily. The former accepted traditional open surgery, while the latter accepted laparoscopic surgery. The operation time, intraoperative blood loss, hospital stay, and time of getting out of bed were compared. The degree of postoperative incision pain was assessed by visual analogue scale (VAS). The life quality was assessed by the Comprehensive Assessment Questionnaire-74 (GQOL-74). The indexes of renal function and urine metabolism were measured. Then, the postoperative stone clearance rate and complications were calculated.

**Results:**

Operation time, blood loss intraoperatively, time out of bed, and hospitalization were all remarkably reduced in the research group, and the difference was statistically significant (*P* < 0.05). The complete stone clearance rates in study and control cohorts were 75.73% and 63.24%, respectively. The VAS scores were lessened after the operation. Compared with the two groups, the VAS scores of the research group were remarkably lower at 1 to 2 weeks and 1 and 3 months after the operation, and the difference was statistically significant (*P* < 0.05). One week after operation, the levels of *β* 2-microglobulin (*β* 2-MG), N-acetyl-*β*-glucosaminidase (NAG), and renal injury molecule-1 (kidney injury molecule-1, Kim-1) in the research group were remarkably lower. The levels of urinary *β* 2-MG, NAG, and KIM-1 in the research group were remarkably lower, and the difference was statistically significant (*P* < 0.05). One week after operation, the levels of urinary oxalic acid, uric acid, and urinary calcium lessened averagely. The levels of urinary oxalic acid, uric acid, and urinary calcium in the research group were lower, and the difference was statistically significant (*P* < 0.05). The quality-of-life scores were compared. One week after the operation, the scores of physical function, psychological function, social function, and material function were all augmented, and the difference was statistically significant (*P* < 0.05). The incidence of complications was 9.56% and 2.21%, respectively. The incidence of complications in the research group was lower, and the difference was statistically significant (*P* < 0.05).

**Conclusion:**

Laparoscopic surgery is successful when treating CRC, which is superior to invasive surgery in postoperative complications, stone clearance rate, improvement of postoperative renal function, and life quality. It is one of the ideal treatment methods for CRC. However, the role of open surgery when treating CRC cannot be ignored. This needs to be further confirmed by large samples of randomized controlled trials.

## 1. Introduction

Urinary calculi are a kind of global disease, which is also one of the most common urological diseases in China. In 1983, it had risen to 86%, and its new incidence was still rising in recent years [1, 2].

Among the main causes of renal stone disease is the abnormal accumulation of crystal substances such as uric acid and oxalic acid in the kidney of the patient. When the accumulation of kidney stones is small, patients can expel them from the body by drinking a lot of water. However, patients are usually unable to detect them effectively in the early stage of the disease. They often wait until the accumulation of kidney stones is too large, and the patients feel obviously uncomfortable [3, 4]. The main incidence group of kidney stone is young and middle-aged male [5]. However, the incidence of kidney stone in male group is much higher than that in female group [6, 7]. For this kind of patients, the stones in the body are mainly removed by operation, while the patients with complex kidney stones are mostly treated by open surgery.

In recent 30 years, with the clinical application of extracorporeal shock wave lithotripsy (ESWL) and percutaneous nephrolithotripsy (PCNL), great changes have taken place when treating renal calculi. Surgery has been remarkably reduced. In spite of this, complex renal stones remain a difficult challenge. Some literature has reported in the world have confirmed that these minimally invasive techniques can still cause varying degrees of renal function damage and have a very high stone residual rate [8]. Surgical treatment is still needed for those cases whose ESWL treatment fails but PCNL and ureteroscopy are not suitable for treatment [9]. Based on the above reality, many scholars have been trying to use laparoscopy to treat upper urinary tract calculi to replace the traditional open surgery to achieve a safe, effective, less pain, and rapid recovery of minimally invasive purpose. Minimally invasive decompressive surgical techniques have excellent results in preserving renal function in management of EPN. The presence of risk factors may not always be associated with high mortality if the patients are treated aggressively in the initial phase of management with minimally invasive techniques. Extracorporeal shock wave is a procedure to break up stones inside the urinary tract, bile ducts, or pancreatic duct with a series of shock waves generated by a machine. The shock waves enter the body and are targeted using an X-ray. Surgery has become the preferred treatment modality for patients with large renal calculi. The technique provides excellent stone clearance, but complication rates are higher than those of minimally invasive techniques, such as ureteroscopy and shock wave lithotripsy. Surgery is still needed for those cases whose ESWL treatment fails, but PCNL and ureteroscopy are not suitable for treatment. Since the 1990s, many scholars at home and abroad began to try to use laparoscopy to treat CRC to replace the traditional open surgery to achieve safe, effective, less pain, and rapid recovery of minimally invasive.

At present, laparoscopic surgery is often used in the clinical treatment of CRC. Although traditional open surgery is less and less, its therapeutic value cannot be ignored. There is no conclusion as to whether this kind of patients should choose traditional open surgery or laparoscopic surgery. At present, the research on the treatment of complex stones by traditional open surgery and laparoscopic surgery mainly would focus on the removal of renal stones and postoperative complications, while neglecting the comparison of patients' life quality. This study was conducted to determine the effectiveness of laparoscopic surgery and traditional open surgery on stone clearance, laboratory indexes, and life quality in patients with renal calculi.

## 2. Patients and Methods

### 2.1. General Information

During March 2017 to March 2022, 272 patients with CRC cured in our hospital were arbitrarily assigned into control group (*n* = 136) and research group (*n* = 136). The former accepted traditional open surgery, while the latter accepted laparoscopic surgery. The control group consisted of patients with ages ranging from 21 to 69, with an average age of 45.83 ± 4.23 years. The control cohort included 73 men and 63 women, and the course of disease ranged from 6 months to 13 years (mean 6.43 ± 1.42) years. Stone distribution was that left 70 cases and right 66 cases. Stone diameter was 2.79 ± 0.61 cm. Stone types were staghorn in 44 cases, complete cast in 40 cases, and incomplete cast in 52 cases. Patients in the research group ranged in age from 27 to 70 years old with an average age of 46.21 ± 4.46. There were 75 men and 61 women, and the course of disease ranged from 7 months to 12 years with an average of (6.32 ± 1.19) years. 67 stones were located on the left side, and 69 stones were located on the right side. The stone diameter is (2.81 ± 0.63 cm). 47 cases were staghorn stones, 39 cases were completely calcified stones, and 50 cases were incompletely calcified stones. General patient data did not show any statistical significance (*P* > 0.05). This study was permitted by the Medical Ethics Council of our hospital, and all patients signed the informed consent form for the trial.

Diagnostic criteria of CRC: All the selected cases were diagnosed as CRC by B-ultrasound, CT, intravenous urography, and hematuria routine examination. The specific diagnostic criteria referred to the guidelines to diagnose and treat urinary calculi [10].

Selection criteria are as follows: (1) all the patients were diagnosed with CRC; (2) there were no cognitive, language, or intellectual impairments, and the patients' basic reading and writing skills were intact, aged ≥18 years old; (3) the clinical data, medical history, and examination records of the patients were perfect; (4) the patients agreed to receive continuous postoperative follow-up and be able to accept and answer telephone follow-up; and (5) in accordance with the indication of operation and anesthesia. Anesthesia indications were absence of lumbar disease and systemic infection. Surgical indications are as follows: stone diameter ≥1.0 cm; stone diameter less than 1 cm, but accompanied by obvious obstruction, hydronephrosis, renal insufficiency, infection caused by stone, and could not be controlled by drugs; and after more than 3 months of conservative treatment, the effect was still not obvious. The above indicators only needed to meet one item to determine the existence of surgical indications.

Exclusion criteria are as follows: (1) patients with serious heart, liver, renal insufficiency, and malignant tumors; (2) patients with coagulation dysfunction; (3) those who refused to participate in the test; (4) patients with renal dysfunction and severe hydronephrosis, urethral or ureteral malformations, and organic urinary tract obstruction; (5) patients with basic diseases affecting the operation; (6) patients with mental diseases; and (7) those who were treated with anticoagulants for a long time.

### 2.2. Treatment Methods

#### 2.2.1. Preoperative Preparation

The day before operation, patients were instructed to undergo general examination, including blood biochemistry, blood lipids, blood glucose, blood coagulation, electrocardiogram, chest plain film, and blood type. Patients over 60 years old were examined by preoperative pulmonary function and cardiac color ultrasound, those with respiratory diseases were examined before operation, and those with cardiovascular diseases were examined by cardiac color ultrasound. Before operation, urinary tract infection was controlled by antibiotics. The day before the operation, the patients were told to eat a small residue diet and given a slow bay agent to empty the intestines. Gastric tube was placed before operation, and gastrointestinal decompression was performed. Catheter was placed to avoid bladder expansion.

#### 2.2.2. Treatment Methods

The control group received traditional invasive surgery. The open lithotripsy was divided into intrarenal sinus pyelolithotomy and pyelolithotomy. The intrarenal sinus pyelolithotomy and surgical incision were made between the 11 intercostals to dissociate the kidney and dissociate along the ureter to the renal hilum until the renal pelvis was found. The research group was treated with laparoscopic nephrolithotomy, including laparoscopic pyelolithotomy, laparoscopic pyelolithotomy, laparoscopic pyelolithotomy, and laparoscopic partial nephrectomy.

(1) Laparoscopic pyelolithotomy or intrarenal sinus pyelolithotomy. Under general anesthesia, all patients were positioned on their contralateral side with an indwelling catheter and lying 90 degrees. To establish pneumoperitoneum, trocar was performed at the umbilical margin or the lateral margin of the rectus abdominis muscle, the anterior line of the umbilical axilla, and the costal edge of the middle line of the clavicle, respectively. The lateral peritoneum and perirenal fascia were opened. During this procedure, the inferior pole of the kidney was exposed, and the renal pelvis and even the renal sinus were separated. After the location of the stone was found, the renal pelvis was longitudinally cut or extended to the intrarenal sinus. The renal pelvis incision was enlarged, and the stone was removed. The renal pelvis and calyx were washed out, and no stone was flushed out. The 4-0 absorbable line of Dmur J tube was placed to suture the renal pelvis incision (the intrarenal pelvis was not sutured), and the perirenal drainage tube was placed to end the operation

(2) Laparoscopic pyelolithoplasty and lithotomy. The operation was performed under general anesthesia, and routine indwelling catheterization was performed before operation. The patient took 90° recumbent position on the healthy side and established pneumoperitoneum. 10-mm and 5-mm cannula needles of diameter were put at the umbilical margin, the anterior axillary line, and the midline of the clavicle. According to the need of the operation, one subcostal incision of the posterior axillary line was added, and the 5-mm trocar was placed. The narrow segments of the UPJ were resected after the kidney, and renal pelvis and ureter were exposed. The ureter was longitudinally opened to 0.5 cm-0.8 cm. The dilated renal pelvis was trimmed, and the calculi in the renal pelvis and calyceal were removed.

The renal pelvis and ureteral incision were closed end-to-end with interrupted sutures of 5-0 or 4-0 absorbable thread. The incision was then restored, and the double J tube with guidewire was put into the peritoneal cavity, the ureter was inserted downwards, and the guidewire is removed. The upper end of the double J-tube was fed into the renal pelvis, and the anterior incision was then interrupted with sutures. The modified renal pelvis incision was sutured continuously with 5-0 or 4-0 absorbable thread, the wound was washed, the perirenal drainage tube was placed, and the operation was ended.

(3) Laparoscopic partial nephrectomy and lithotomy. The patient received general anesthesia, routine indwelling catheterization before operation, and 90-degree healthy lateral position. 10-mm and 5-mm cannulas of diameter were put at the umbilical margin, the anterior axillary line, and the midline of the clavicle. If necessary, the 5 mm cannula was used to expose the kidney. In addition, 1 cm-diameter cannula with a diameter of 1 cm was worn at the posterior lower part of the endoscopic cannula to place a noninvasive intestinal forceps that controlled the renal pedicle vessels. During the operation, the lateral peritoneum and perirenal fascia were opened. The renal pedicle and the middle and inferior pole of the kidney were dissociated and exposed to fully control the renal pedicle and facilitate the removal of the inferior pole of the kidney and the treatment of the wound. The specimen bag and suture equipment were prepared. The wound was sutured with 2-0 absorbable line\ “8\” or continuous suture to stop bleeding. When the blocking time of renal pedicle reached 25 min, the renal pedicle forceps were opened about 1 min~2 min (in 2 cases of renal ischemia 25 min, only the forceps were opened once, and only the forceps were opened without removing the renal pedicle clamp), and then reclamped to control the renal pedicle to continue to deal with the wound. After the wound was closed, an attempt was made to open the renal infarct noninvasive bowel clamp. If there was bleeding, suture the bleeding site with the word “8\” to stop the bleeding. If the operative field was not clear, the renal pedicle could be reclamped to control the renal pedicle and then suture to stop the bleeding. When there was no bleeding in the incision, the renal pedicle noninvasive intestinal clamp was removed. The operation was finished by releasing the skin tube around the kidney.

### 2.3. Observation Index

#### 2.3.1. Operation Related Index

In addition to intraoperative blood loss, operating time, postoperative hospital stays, time spent out of bed, and stone clearance rate, we calculated postoperative complications. Amount of blood lost intraoperatively is the amount of blood lost during the surgery. Stone clearance rate = (the number of cases meeting the stone clearance criteria/the total number of cases in this group) × 100%. Approximately one month after their operations, each patient was followed up. The number of complications like urinary fistula, incision infection, bleeding, ureteral injury, renal function injury, and other complications were statistically compared. The incidence of complications = (sum of all kinds of complications/total number of cases in this group) × 100%. The operation time was the difference between patients going in and out of the operating room. Postoperative hospital stay referred to the time from the completion of the operation to the discharge of the patient. The time to get out of bed referred to the time it takes from the end of the operation to the first time to get out of bed. The stone clearance rate was recorded and analyzed when the patient was discharged [11].

#### 2.3.2. VAS Scoring

VAS score was employed to measure the pain degree before and after operation, and the full score was 10. The specific evaluation criteria were as follows: 0: no pain; <3: mild pain, bearable; 4-6: pain and affect sleep; and 7-10: strong pain, unbearable, and affecting life. The patients were evaluated before treatment, 1 to 2 weeks, and 1 and 3 months after operation.

#### 2.3.3. Renal Function and Urinary Metabolic Index

The second 4-7 mL of morning urine was obtained before and 1 week after operation. The levels of *β* 2-MG, NAG, and Kim-1 were analyzed by enzyme-linked immunosorbent assay (Elisa) on Beckman BS-460. Urinary metabolic indexes, including urinary oxalic acid, uric acid, and urinary calcium, were measured by automatic analyzer.

#### 2.3.4. Life Quality Score

The life quality of the patients was evaluated with the life technician GQOL-74 [12] before and 1 week after operation. The scale involved four aspects, including physical, psychological, social, and material function.

### 2.4. Statistical Analysis

IBMSPSS24.0 software was applied for statistical analysis. The measurement data were expressed by mean ± standard deviation. The counting data were expressed by frequency or rate. *T*-test was used when measurement data obey normal distribution, and rank sum test was used when it did not obey normal distribution. *χ*2 test was used to compare the classified counting data. Repeated measurement data were analyzed by repeated measurement analysis of variance. The main effect test results were used when there was no interaction, and simple effect analysis was carried out when there was interaction. *P* < 0.05 indicated that the difference between groups is statistically significant.

## 3. Results

### 3.1. Surgical Indexes

Operation time, blood loss intraoperatively, time out of bed, and hospitalization are all remarkably reduced in the research group, and the difference is statistically significant (*P* < 0.05), as indicated in Table 1.

### 3.2. Stone Clearance Rate

In the comparison of stone clearance rate, 103 cases were completely removed, 23 cases were slightly residual, and 10 cases were obvious residual. The complete stone clearance rate was 75.73% in the research group. While 86 cases, 37 cases and 13 cases in the control group were completely removed. The complete stone clearance rate was 63.24%. Compared between groups, the complete stone clearance rate in the research group is higher, and the difference is statistically significant (*P* < 0.05), as indicated in Figure 1.

### 3.3. VAS Score Comparison

Repeated measures analysis of variance found that there exhibited a statistically remarkable difference in the VAS score (*P* < 0.05). There exhibited remarkable difference among different time points (*P* < 0.05). There exhibited remarkable difference in × time interaction, and the difference was statistically significant (*P* < 0.05). After treatment, the VAS scores were lessened. VAS scores of the research group are remarkably lower at 1 to 2 weeks and 1 and 3 months after the operation, and the difference is statistically significant (*P* < 0.05), as indicated in Table 2.

### 3.4. The Renal Function Indexes

One week after the operation, the levels of *β* 2-MG, NAG, and KIM-1 were lessened. Compared with the two groups, the levels of which in the urine of the research group are remarkably lower one week after the operation, and the difference is statistically significant (*P* < 0.05), as indicated in Table 3.

### 3.5. The Urine Metabolism

One week after operation, the levels of urinary oxalic acid, uric acid, and urinary calcium lessened averagely. Compared with the control group, the levels of urinary oxalic acid, uric acid, and calcium in the research group are remarkably lower, and the difference is statistically significant (*P* < 0.05), as indicated in Table 4.

### 3.6. The Quality-of-Life Scores between the Two Groups

One week after the operation, the physical, psychological, function, and material function scores were augmented. Compared with the two groups, the physical, psychological, social, and material function scores of the research group are higher, and the difference is statistically significant (*P* < 0.05), as indicated in Table 5.

### 3.7. The Incidence of Postoperative Complications

In the control group, there were 5 cases of urinary fistula, 1 case of incision infection, 3 cases of bleeding, 1 case of ureteral injury, and 3 cases of renal function injury. The incidence of complications was 9.56%. In the research group, urinary fistula, incision infection, and renal function injury occurred in 1 case, and the incidence rate of postoperative complications was 2.21%. The incidence of complications in the research group is lower, and the difference is statistically significant (*P* < 0.05), as indicated in Figure 2.

## 4. Discussion

The treatment of complex kidney stones is still a difficult problem at present. PCNL is considered to be the best choice to treat these stones [13]. However, not all cases are suitable for PCNL treatment [14, 15]. At the same time, complications such as massive hemorrhage, severe injury, and intrarenal infection after PCNL treatment still limit the application of PCNL [16]. Nowadays, the pathogenesis of renal calculi is not fully understood, which may be relevant to heredity, metabolism, infection, environment, diet, anatomy, and drugs. Among them, complex renal stones refer to stones whose diameter is longer than 2.5 cm, staghorn calculi, multiple stones, and difficult to remove stones due to abnormal renal function or anatomy [16–18]. Because this operation is required high experience and skills of laparoscopic surgery, many urologists prefer ESWL, PCNL, and traditional open surgery to treat CRC [19]. Laparoscopic surgery, however, is more readily apparent when compared with traditional open surgery in minimally invasive surgery.

We showed that laparoscopic surgery spent less time, less blood loss, and faster postoperative recovery than traditional open surgery, which fully confirmed the safety of laparoscopic surgery in this study. The application of laparoscopic surgery can also effectively reduce the postoperative stone residual rate and improve the stone clearance rate in patients with CRC, which can prove that the operation has a remarkable clinical efficacy and safety to treat CRC. In this study, the VAS scores of patients with laparoscopic surgery at 1 to 2 weeks and 1 and 3 months after operation were lower than those with traditional open surgery. It was mainly because laparoscopic surgery was a minimally invasive operation with small incision, less damage to normal tissue, and lower risk of various complications; the postoperative recovery was faster; and the pain symptoms of patients were milder. This study was conducted to determine the effectiveness of laparoscopic surgery and traditional open surgery on stone clearance, laboratory indexes, and life quality in patients with renal calculi.

The common clinical complex renal stones are staghorn calculi and intrapelvic cast stones [20]. For single branch staghorn calculi of extrarenal renal pelvis or complete intrapelvic cast stones, laparoscopic pyelolithotomy can be performed successfully. However, for intrarenal pyelolithiasis, staghorn calculi with multiple branches growing into different calyceal and multiple calyceal stones with secondary infundibulum stenosis or calyceal diverticulum, it is much more complicated, and laparoscopic pyelolithotomy alone may not be successful. Currently, intrarenal sinus peotomy or partial renal parenchyma incision becomes necessary [21, 22].

It was very important for the smooth removal of staghorn stones, because this approach can make it easier for us to separate to the funnel part. For staghorn stones with multiple branches, only the shorter branch of the lower calyx was delivered out of the renal pelvis, and the longer branch of the upper calyx was successfully removed. The experience of Rhudd AR is worth using for reference. In our study, most laparoscopic pyelolithotomy was performed through laparoscopic pyelolithotomy (including intrarenal sinus pyelolithotomy). For laparoscopic pyelolithotomy, good exposure is the key to successful operation, while transabdominal approach is easier to expose the kidney and separate renal pelvis 137, so transabdominal approach is used in our study. During the operation, the middle and inferior pole of the kidney should be freed as much as possible, and the inferior pole of the kidney should be raised or gauze padded into the inferior pole of the kidney to expose the kidney. Blunt or sharp separation can be chosen when separating the renal pelvis, but it must be noted that the action of separation should be patient and skillful. Sometimes, due to the serious adhesion of the surrounding tissue, separation will be very difficult and easy to bleed, which requires more patience and meticulous, and the selection of electrocoagulation hook separation will help to separate, especially when separating the renal pelvis in the renal sinus. According to the experience of Radfar MH et al. electrocoagulation hook was selected to separate. The direction of separation was more precise and accurate, and small vascular bleeding affecting the visual field of operation can also be found immediately. Moreover, electrocoagulation can be used to stop bleeding [23]. When cutting and removing stones, the incision should be above the stones, and the incision should be large enough to facilitate the removal of stones, especially upward as far as possible into the renal sinus. However, it should not go beyond the junction of the renal pelvis and ureter so that the ureter was not torn during subsequent examination of the calyces and the removal of the stone. Loosening and removing stones was also a very patient and skillful task, especially for more branched staghorn stones. YanQ et al. introduced that when loosening and peeling off stones [24], we should start from the right side of the stones [24].

*β* 2-MG can moderate small molecule globulin, can reflect the degree of glomerular injury, and has high specificity and sensitivity [25]. KIM-1 was highly expressed in hypoxic renal tissue, and its level was relevant with the degree of renal tubular injury positively [26]. NAG is a marker of lysosomes, which is very abundant in renal tubular epithelial cells. When the glomerular filtration membrane is damaged, NAG can enter the urine, causing the level of urinary NAG to increase. This research showed that compared with traditional surgical treatment, laparoscopic treatment could reduce the damage of renal tissue in patients with renal calculi to some extent and protect renal function. The analysis of the reason was that laparoscopic surgery can decide the specific location, size, shape, and number of stones on the premise of avoiding great trauma caused by traditional laparotomy and remove the stone thoroughly and effectively. At the same time, ultrasonic knife resection of adhesive tissue can effectively stop bleeding and further reduce the amount of bleeding during operation. The laparoscopy has three-dimensional visual effect, which can enlarge the image. For larger stones or incarcerated stones, we can choose the clamp method to remove the stones according to the actual situation. It is beneficial to the thorough removal of stones and reduce the occurrence of residual stones. During the period of renal stone lithotripsy, in order to ensure that the surgical field is clearly visible, a large amount of water needs to be irrigated through the working channel. However, the water perfusion pressure is higher than the physiological pressure in the renal pelvis, and it is simple to cause urinary reflux in the renal pelvis and damage renal tissue.

Laparoscopic surgery is difficult to operate, which requires higher hardware equipment. In addition, the cost of hospitalization is higher than that of open surgery, which limits the wide development of laparoscopic surgery. After the removal of urinary calculi, the urinary tract was unobstructed, hydronephrosis was gradually relieved, and the life quality and anxiety were improved. This study was also indicated that laparoscopic surgery was better than traditional surgery in these three aspects. The reason may be that long-term surgical posture has an adverse effect on the comfort of patients, which may affect the late recovery of patients [27]. In addition, laparoscopic surgery has fewer complications than traditional surgery, which is also one of the reasons for the high life quality of patients. Minimally invasive decompression surgery techniques have been shown to be effective in preserving renal function in EPN. The presence of risk factors is not necessarily associated with high mortality if the patient is treated aggressively with minimally invasive techniques in the initial stages of management. Extracorporeal shock wave is a procedure in which a series of shock waves generated by a machine is used to break up the urinary tract. The shock waves enter the body and are located using X-rays. The procedure has become the treatment of choice for patients with large kidney stones. The technique provides good stone removal but has a higher complication rate than minimally invasive techniques such as ureteroscopy and shock wave lithotripsy. This study still has some shortcomings. Firstly, the quality of this study is limited due to the small sample size we included in the study. Secondly, this research is a single-center study, and our findings are subject to some degree of bias. Therefore, our results may differ from those of large-scale multicenter studies from other academic institutes. This research is still clinically significant, and further in-depth investigations will be carried out in the future.

To sum up, laparoscopic surgery has a higher application value in patients with renal stone diseases, with remarkable advantages such as less trauma, high safety, high stone clearance rate, and protection of renal function, which can remarkably enhance the postoperative life quality of patients.

## Figures and Tables

**Figure 1:** Stone clearance rate between the two groups.

**Figure 2:** Comparison of postoperative complications between the two groups.

**Table 1:** The surgical indexes between the two groups $\left[\bar{x}\pm s\right]$.

Grouping	*N*	Operation time (min)	Intraoperative bleeding volume (mL)	Time to get out of bed (d)	Hospitalization time (d)
Control group	136	153.38 ± 12.45	253.18 ± 14.22	3.25 ± 0.64	12.46 ± 2.63
Research group	136	121.42 ± 10.53	97.25 ± 10.08	1.67 ± 0.28	7.52 ± 1.17
*t* *value*		22.858	104.327	26.376	20.104
*Pvalue*		<0.05	<0.05	<0.05	<0.05

**Table 2:** The postoperative VAS scores between the two groups [*x̅*±*s*, points].

Grouping	*N*	Before treatment	One week after operation	2 weeks after operation	One month after operation	Three months after operation
Control group	136	6.42 ± 2.17	4.72 ± 1.91	3.14 ± 0.42	1.08 ± 0.14	0.92 ± 0.14
Research group	136	6.33 ± 2.06	3.42 ± 1.23	1.83 ± 0.87	0.89 ± 0.03	0.33 ± 0.06
Intergroup (F/P)	39.662/0.000					
Time (F/P)	51.846/0.000					
Intergroup × time (F/P)	60.091/0.000					

**Table 3:** The urinary *β* 2-MG, NAG, and KIM-1 levels between the two groups after operation $\left[\bar{x}\pm s\right]$.

Grouping	*N*	*β* 2-MG (mg/L)		NAG (IU/L)		KIM-1 (ng)	
		Before operation	One week after operation	Before operation	One week after operation	Before operation	One week after operation
Control group	136	0.45 ± 0.18	0.36 ± 0.07^a^	9.06 ± 1.83	7.28 ± 1.63^a^	91.24 ± 9.53	84.83 ± 8.27^a^
Research group	136	0.48 ± 0.15	0.21 ± 0.05^b^	9.22 ± 1.76	5.84 ± 1.66^b^	90.09 ± 9.41	77.63 ± 7.84^b^
*tvalue*		1.493	20.335	0.735	7.218	1.001	7.368
*Pvalue*		>0.05	<0.05	>0.05	<0.05	>0.05	<0.05

Note: The comparison between the control group before and after operation, ^a^*P* < 0.05. The comparison of preoperative and postoperative in the research group, ^b^*P* < 0.05.

**Table 4:** The urine metabolism between the two groups $\left[\bar{x}\pm s\right]$.

Grouping	*N*	Urinary oxalic acid (mmol/L)		Uric acid (mmol/L)		Urinary calcium (mmol/L)	
		Before operation	One week after operation	Before operation	One week after operation	Before operation	One week after operation
Control group	136	5.82 ± 0.38	3.62 ± 0.23	0.71 ± 0.23	0.49 ± 0.01	6.36 ± 1.83	4.19 ± 0.83
Research group	136	5.77 ± 0.35	2.68 ± 0.17	0.78 ± 0.29	0.27 ± 0.03	6.73 ± 1.65	3.06 ± 0.45
*tvalue*		0.129	38.328	2.206	81.132	1.751	13.958
*Pvalue*		>0.05	<0.05	>0.05	<0.05	>0.05	<0.05

Note: The comparison between the control group before and after operation, ^a^*P* < 0.05. The comparison of preoperative and postoperative in the research group, ^b^*P* < 0.05.

**Table 5:** The quality-of-life scores between the two groups [*x̅*±*s*, points].

Grouping	*N*	Somatic function		Psychological function		Social function		Material function	
		Before operation	One week after operation	Before operation	One week after operation	Before operation	One week after operation	Before operation	One week after operation
Control group	136	51.89 ± 10.36	63.66 ± 10.45^a^	52.56 ± 12.48	65.23 ± 15.48^a^	63.57 ± 8.15	79.83 ± 3.56^a^	57.83 ± 8.46	81.37 ± 18.79^a^
Research group	136	52.34 ± 11.37	78.89 ± 16.23^b^	52.36 ± 12.44	79.35 ± 15.41^b^	61.93 ± 8.43	71.03 ± 12.15^b^	58.61 ± 7.46	66.84 ± 4.83^b^
*tvalue*		0.341	9.201	0.132	7.539	1.631	7.176	0.806	8.734
*Pvalue*		>0.05	<0.05	>0.05	<0.05	>0.05	<0.05	>0.05	<0.05

Note: The comparison between the control group before and after operation, ^a^*P* < 0.05. The comparison of preoperative and postoperative in the research group, ^b^*P* < 0.05.

## Data Availability

The datasets used and analyzed during the current study are available from the corresponding author upon reasonable request.
